# Research on the Improved CNN Deep Learning Method for Motion Intention Recognition of Dynamic Lower Limb Prosthesis

This article has been retracted.

**DOI:** 10.1155/2021/7331692

**Published:** 2021-12-06

**Authors:** Qiulin Wang

**Affiliations:** Yangzhou University, Yangzhou 225000, China

## Abstract

**Objective:**

In order to study the motion recognition intention of lower limb prosthesis based on the CNN deep learning algorithm.

**Methods:**

A convolutional neural network (CNN) model was established to reconstruct the motion pattern. Before the movement mode of the affected side was converted, the sensor was bound to the healthy side. The classifier was employed to extract and classify the features, so as to realize the accurate description of the movement intention of the disabled.

**Results:**

The method proposed in this research can achieve 98.2% recognition rate of the movement intention of patients with lower limb amputation under different terrains, and the recognition rate can reach 97% after the pattern converted between the five modes was added.

**Conclusion:**

The deep learning algorithm that automatically recognized and extracted features can effectively improve the control performance on the intelligent lower limb prosthesis and realize the natural and seamless conversion of the intelligent prosthesis in a variety of motion modes.

## 1. Introduction

The results of the national sample survey of disabled persons indicated that the number of physically disabled persons in China was close to more than 25 million, which was about 6.34%. In this survey, the number of amputees alone accounted for 70% of the total number of amputees. Due to various uncertain and unexpected factors in life such as diseases, natural disasters, traffic accidents, and birth defects, the number and proportion of lower limb amputations are still rising for many reasons, so the research on lower limb prostheses is particularly important [1–3]. Different from the disability of the upper limb, the lower limb prosthesis is directly related to the balance of human motion, which very directly affects the life and psychological state of the patient [4]. The adoption of mechanical prostheses brings inconvenience to the life of patients to a certain extent, and patient cannot easily walk on complex terrain, such as up and downstairs. Even on a flat ground, the metabolic energy of the patient's body is 60% higher than that of the healthy subject. Therefore, to solve the limitations of this mechanical prosthesis, the researchers started the research on the intelligent power lower limb prosthesis [5]. The movement of the lower limbs is a complex movement, but the movement of the lower limbs also has certain regularity and periodicity. The adoption of appropriate sensors to obtain human movement and physiological information has become a prerequisite for intelligent prosthetic control [6]. The existing international information source for lower limb prosthesis control is physical quantities related to motion information. Such kind of information can directly reflect the biological characteristics of human movement, and the collection is relatively simple, and it is particularly suitable for implementing control. Now, smart lower limb value products adopt one or more sensors to measure human movement information according to different control methods [7].

According to the difference of the collected signals, the intention recognition of the lower limb prosthesis is classified into the following types: those based on the biomechanical signal, those based on the bioelectric signal, and the intention recognition of fusion of various types of data [8]. However, the traditional recognition methods of motion intention have many shallow learning methods based on machine learning and pattern discrimination. Feature extraction is mainly manual extraction, such as maximum value, minimum value, correlation coefficient, and standard deviation [9]. The selection of classifiers is based on data types and feature attributes, such as support vector machines, dynamic Bayesian networks, and linear discriminant analysis.

Human movement intention recognition plays a very important role in the research of intelligent lower limb prosthetics, for it will give a safe, free, and seamless period of relief between exercise modes. In the study of lower limb prosthetic intention recognition, there are many difficulties, such as sensor selection and fusion, data classification algorithm, and control strategy [10]. Some researchers obtained the patient's motion diagram by extracting the electrical signals of the residual muscle in the thigh. There were also researchers who put the sensor on the healthy side of the new strategy, which solved the problem of lag in the recognition of movement intentions [11]. Many domestic and foreign research reports indicated that machine learning algorithms had achieved good classification results in the recognition of lower limb prosthetic movements. Most researchers mainly adopted classifiers such as SVM, hidden Markov, decision tree, and template matching [12].

## 2. Methods

### 2.1. Introduction to Gait Cycle

According to the periodicity of the lower limbs, in the same gait pattern, the movement of the lower limbs is divided into multiple gait cycles. According to the regularity of the alternating contact between the feet and the ground, it is divided into two gait events: toes off the ground and heels on the ground. For this reason, the gait cycle is divided into two main phases, the support phase and the swing phase, as shown in Figure 1.

### 2.2. Sport Mode

Walking in daily life is one of the most common and regular movements of the lower limbs of the human body, and it is also one of the key features that distinguish humans from other animals. The normal gait of a person when walking does not requires thinking; it is completed through the coordinated movement of the hip, knee, and ankle joints. The torso is basically kept on the supporting surface between the feet. Starting from the law of gait, the movement mode has the most basic level walking, uphill, downhill, upstairs, and downstairs. The modes of transformation in life include flat to uphill, downhill, upstairs, downstairs, uphill to flat walking, downhill to flat walking, upstairs to flat walking, and downstairs to flat walking; walking steadily on level ground; and steadily go up the stairs, go down the stairs steadily, go uphill steadily, and go downhill steadily. In the normal pace of a healthy person, the duration of the dual support period is inversely proportional to the walking speed. The exercise phase includes the single-leg support phase (SS) and the flight phase (flight). When a person is walking, the empirical equation for the time and frequency of the legs is as follows.

(1) $$\begin{array}{c} Y_{ds}=\frac{\left(-0.16p+29.08\right)\cdot t_{p}}{100}. \end{array}$$

*Y*_*ds*_ represents the time of the bipedal support period, *t*_*p*_ represents the walking cycle, and *p* represents the walking frequency. When *p* increases to a certain extent, it transitions from walking to running.

In this research, the sensor was placed on the healthy side of the patient. The first type of the transition step starts at the moment when the toe of the previous foot is off the ground under the previous terrain condition. It ends when the heel of the same foot hits the ground and the next terrain. There are also special situations in walking, such as switching from level ground to upstairs and downstairs, which requires a new definition. The second type starts at the moment when the toe of the back foot is off the ground under the previous terrain condition and end the ground with the heel of the foot on the same side and the next terrain.

### 2.3. Motion Recognition Flowchart

In Figure 2, it first describes the intent of the object space and then goes to the defined pattern space. Then, the features are extracted in the feature space, and finally, the collection of the type space is acquired.

### 2.4. Convolutional Neural Network

Deep learning is an efficient and unsupervised algorithm technology that can be compared to the human brain, which simulates the behavioral characteristics of the brain to analyze and interpret data. The CNN, as one of many algorithms in depth science, usually consists of *N* feature extraction layers, lower sampling layers, and *N* fully connected classifiers. It has very low model complexity and very few weights. The image can be input without conversion to reduce the complex process of feature extraction. The image input is the bottom layer, and the network can obtain the basic features of the image. In this way, it has good resistance to the deformation and rotation of the target object or image, and it is very effective to take *m* images as the input in the task of computer vision or door recognition.

Figure 3 is the diagram of a CNN. *Y_x* is the convolutional layer, *D_(X* *+* *1)* is the downsampling layer, *E_x* and *G_* are the multiplicative biases, *B_x* is the additive bias, and *ω* is the Sigmoid function.

### 2.5. Construction of the CNN

The CNN has seven layers in the normal state, which are the input layer, convolution layer, subsampling layer, fully connected layer, and output layer. There are many independent neurons distributed on each level. Subsampling will integrate all the features that need to be extracted when extracting features, and then, the fully connected layer will classify these features (Figure 4).

In a CNN, the feature maps of different convolution kernels exist in any convolutional layer, and many independent neurons are distributed on the feature map. Neurons with the same feature map will share a convolution kernel. Any neuron will accept the input information in the domain, then perform convolution processing together with the convolution kernel, and finally obtain the processed feature map.

### 2.6. Data Establishment

In the experimental group, there were 10 subjects recruited, including 8 healthy and 2 disabled with left leg amputation. 8 healthy people included 4 men and 4 women, the height range was 162–180 cm, the weight was 45–80 kg, and the age was 22–35. In daily life, when a normal person encounters going up or down or going up or downhill, whether the left foot or the right foot is taken first, there is a certain degree of randomness. Before switching between different exercise modes, amputees will adjust the step length by themselves based on experience to ensure the safety of the exercise and perform the switching exercise on the healthy side. To simulate the walking habits of lower limb amputees as much as possible, the walking sequence of healthy and amputees should be consistent.

## 3. Results and Analysis

### 3.1. Accuracy

Compared with the recognition in reference [13], the accuracy of A and B (Figure 5) was 94.3% and 95.6%, respectively. The accurate recognition rate in this research was 98.2%, which was significantly higher than the other two methods. In the past, feature extraction was done manually. Compared to traditional methods, the automatic mode was adopted in this research, which effectively reduced the interval delay in the manual mode, with higher utilization and greater accuracy.

### 3.2. Movement Mode Confusion Matrix

In Figure 6, the average recognition rate of the five steady-state modes was 97.8%. The recognition effect of downhill was relatively poor. 2% of the samples were recognized as walking parallel, 2% were recognized as going downstairs, and 2% of the samples walking parallel were identified as going downstairs. The recognition effect of going downstairs and going upstairs was good, for only 1% of the samples was not accurate. 1% of going upstairs was recognized as going downstairs, and 1% of going downstairs was recognized as going upstairs. 3% of uphill were recognized as downhills. It was obvious that the accuracy on both the uphill and downhill had a large lifting space.

## 4. Discussion

The traditional way of motion intention recognition is mainly to embed sensors on the prosthesis and extract some features during mode conversion during walking. The data of the swing phase of the sensor in the conversion step are collected, which are then analyzed. During the transition step, it takes on a different movement gait between the front and the back, which causes a delay in the sensors on the prosthesis. If the data collected in this way arre adopted, there will be inaccuracy and lagging shortcomings. Furthermore, the recognition of motion intention by the sensor and the control of the lower limb prosthesis will definitely have a certain delay, and it will not be able to fully reflect the real motion intention recognition. This research broke the previous traditional model, adopted a single inertial sensor to collect the early data of the swing phase state on the healthy side, and then utilized the constructed CNN for identification [14]. After the movement intention of the healthy side was recognized, the symmetric mapping relationship was adopted to identify the movement intention of the affected side. The prosthetic controller accepted the recognition results passed to it in advance and adjusted the controlled parameters in time during this process. This approach avoided the shortcomings of obvious hysteresis, allowed the disabled to transition to the next movement state naturally and smoothly, and ultimately achieved true intention recognition.

## 5. Conclusion

Based on the CNN deep learning model, the motion intention of the intelligent lower limb prosthesis was recognized, and a network neural network was built. The motion parameters in the prosthetic motion mode were adjusted in time, and the deep features of the data were automatically extracted. The delay problem of traditional manual recognition was solved, and the motion intention of the prosthesis was also truly recognized. Compared with other research methods, the accuracy of the CNN algorithm was higher, which provided a basis for helping the disabled achieve stable and smooth walking. However, the recognition of the model in this research cannot reach 100% for each category, which will be the focus of the next research.

## Figures and Tables

**Figure 1:** Schematic diagram of human gait.

**Figure 2:** General flowchart of motion intention recognition.

**Figure 3:** Schematic diagram of CNN structure.

**Figure 4:** Schematic diagram of CNN structure.

**Figure 5:** Accuracy comparison.

**Figure 6:** Confusion matrixes of five steady-state modes.

## Data Availability

The data used to support the findings of this study are available from the corresponding author upon request.
